The article "Evaluation and comparison of the efficacy and safety of cross‐linked and non‐cross‐linked hyaluronic acid in combination with botulinum toxin type A in the treatment of atrophic acne scars: A double‐blind randomized clinical trial" was published in 2024. Journal: Skin Res Technol.

# Evaluation and comparison of the efficacy and safety of cross‐linked and non‐cross‐linked hyaluronic acid in combination with botulinum toxin type A in the treatment of atrophic acne scars: A double‐blind randomized clinical trial

**DOI:** 10.1111/srt.13541

**Published:** 2024-01-04

**Authors:** Elham Behrangi, Abbas Dehghani, Farzad Sheikhzadeh, Azadeh Goodarzi, Masoomeh Roohaninasab

**Affiliations:** ^1^ Department of Dermatology Rasool Akram Medical Complex Clinical Research Development Center (RCRDC) School of Medicine Iran University of Medical Sciences (IUMS) Tehran Iran; ^2^ School of Medicine Iran University of Medical Sciences (IUMS) Tehran Iran

**Keywords:** acne, acne scars, atrophic scar, clinical trial, cross‐linked, efficacy, hyaluronic acid, non‐cross‐linked, safety, scar

## Abstract

**Introduction:**

Acne vulgaris is a common skin condition that affects a significant percentage of adolescents, with scarring being one of its permanent complications. This study aims to compare the efficacy and safety of using botulinum toxin type A (BTA) in combination with cross‐linked and non‐cross‐linked hyaluronic acid (HA) for the treatment of atrophic acne scars.

**Method:**

Our study is a randomized, double‐blind clinical trial conducted on 16 patients with atrophic acne scars. The patients were randomly assigned to one of two groups: one group received a single session of BTA and crossed link HA combination, while the other group received two sessions of BTA and non‐crossed link HA, 1 month apart. The patients were followed up at 3 and 6 months after baseline to evaluate the number and area of fine and large pores and spots, scar grading, patient satisfaction, and complications.

**Results:**

The mean age of individuals in both the cross‐linked HA and non‐cross‐linked HA groups was 32.75 ± 4.26 and 31.50 ± 8.48 years, respectively (*p* = 0.71). In terms of gender, three (37.5%) and seven (87.5%) individuals in the cross‐linked and non‐cross‐linked HA groups were female, respectively (*p* = 0.11). There were no significant differences in the count and area of fine and large pores and spots between the two groups at baseline and the first follow‐up session. However, in the second follow‐up session, the non‐cross‐linked HA group had significantly better results than the cross‐linked HA group in terms of large pores count and area (*p* = 0.01). In terms of changes over time, the non‐cross‐linked HA group showed significantly better improvements in the count and area of large pores compared to the cross‐linked HA group (*p* = 0.03). Additionally, both groups experienced a significant decrease in the count and area of fine pores over time (*p* = 0.001), but the amount of changes was not statistically significant between the two groups (*p* = 0.06). Concerning acne grade, initially, 62.5% and 12.5% of cases in the cross‐linked HA and non‐cross‐linked HA groups, respectively, had severe grades. However, in the last session, these percentages significantly decreased to 0% for both groups (*p* = 0.002 and 0.005, respectively). In terms of treatment complications, none of the patients experienced any adverse effects.

The article "Evaluation and comparison of the efficacy and safety of cross‐linked and non‐cross‐linked hyaluronic acid in combination with botulinum toxin type A in the treatment of atrophic acne scars: A double‐blind randomized clinical trial" was published in 2024. Journal: Skin Res Technol.

**Conclusion:**

The study demonstrated that both cross‐linked HA and non‐cross‐linked HA were effective in reducing acne severity and improving the appearance of pores and spots. The treatments had similar effects on fine pores, spots, and overall acne severity. However, non‐cross‐linked HA appeared to have a better result on large pores compared to cross‐linked HA.

## 1 INTRODUCTION

Acne vulgaris is a common skin condition especially in adolescents affecting 95–100% of boys and 83–85% of girls, and in 12–14% of cases it persists into adulthood.^1^, ^2^ Scar is considered one of the permanent complications of acne, resulting from the destruction of collagen fibers and subcutaneous fat, and affect up to 95% of acne patients, depending on the severity and delay in starting treatment.^3^

The most common form of acne scar is atrophic scar, which is divided into three types: Rolling, Boxcar, and Ice‐pickle, with Ice‐pickle scar accounting for 60–70% of all atrophic scars.^3^, ^4^

The treatment of atrophic acne scars specially icepick types is always challenging for dermatologists, and so far, different methods such as chemical peeling, dermabrasion, needling, subcision, and lasers have been used to treat patients with this type of scars.^1^, ^5^ However, each of the methods has its own limitations, and ultimately, the improvement that results are not satisfactory compared to the cost and time involved, and taking into account the complications. For example, in fractional laser treatment, the patient suffers from severe pain, and the recovery period after treatment is long. In addition, the laser cannot be used to treat active acne because postinflammatory hyperpigmentation remains. Or with microneedling, multiple sessions are required to treat atrophic acne scars.^6^

Hyaluronic acid (HA) is a naturally occurring substance in the body that is found in high concentrations in the skin.^7^ It plays an important role in maintaining skin hydration and elasticity. In recent years, HA has become a popular ingredient in skincare products and cosmetic treatments due to its ability to improve skin texture and reduce the appearance of fine lines and wrinkles^8^. When HA comes to treating acne scars, there are two types that are commonly used: cross‐linked and non‐cross‐linked. Non‐cross‐linked HA is a pure form of the molecule that is not chemically modified. It is often used in topical skincare products to hydrate and plump up the skin.^1^, ^9^ Cross‐linked HA, on the other hand, is modified through a chemical process that creates bonds between the molecules. This makes the HA more resistant to degradation by the body, allowing it to last longer when injected into the skin. Cross‐linked HA is often used in dermal fillers to treat deeper, more severe acne scars.^8^, ^9^

Both types of HA can be effective in reducing the appearance of acne scars, but the choice between cross‐linked and non‐cross‐linked HA will depend on the severity of the scarring and the desired outcome.^9^, ^10^ Cross‐linked HA is used because it provides stability, cohesion, and elasticity to the skin to improve volume and skin texture, and non‐cross‐linked HA is used to treat atrophic acne scars by stimulating collagen production. Cross‐linked HA lasts longer, but treatment with it is much more expensive.^8^, ^11^

For more than 20 years, botulinum toxin has been used in the facial area or outside the face to relax muscles and reduce unnecessary movements. Another application of this toxin is the treatment and prophylaxis of atrophic acne scars. Botulinum toxin reduces the tension of the muscles surrounding the scar.^6^, ^12^, ^13^

One of the new methods in the treatment of atrophic acne scars, for which few studies are available, is the use of cross‐linked and non‐cross‐linked HA in combination with botulinum toxin type A. The aim of this study is to compare the efficacy and safety of the BTA injection in combination with cross‐linked HA and non‐cross‐linked hyaluronic in the treatment of atrophic acne scar.

The article "Evaluation and comparison of the efficacy and safety of cross‐linked and non‐cross‐linked hyaluronic acid in combination with botulinum toxin type A in the treatment of atrophic acne scars: A double‐blind randomized clinical trial" was published in 2024. Journal: Skin Res Technol.

## 2 MATERIALS AND METHODS

### 2.1 Patients

This randomized, double‐blind clinical trial was carried out on 16 patients aged 18–40 years with atrophic acne scars who were referred to a dermatology clinic from February to May 2022. At baseline, patients' background information was collected and entered into the study checklist. For all patients, the baseline examination was performed quantitatively by measuring the count and area of fine pores, large pores, and spots. Patients were then randomly assigned to one of two groups: one group received a single session of the BTA and crossed link HA combination, while the other group received two sessions of the combination of BTA and non‐crossed link HA, 1 month apart.

Patients were informed about the procedures and gave their written consent before the trial began, with the assurance that the procedures would not cause complications or require any costs. Eligible patients were those between 18 and 40 years old with atrophic acne scars who agreed to participate and attend follow‐up appointments. Patients with active acne, inflammation or infection at the procedure site, severe internal disease, concomitant disease at the treatment site, platelet dysfunction or thrombocytopenia, and those who had used anticoagulants or NSAIDs within the past 48 h were excluded from participation.

### 2.2 Randomization and blinding

The study involved patients who were divided into two intervention groups using a randomized list. The groups received either a combination injection of BTA and crossed link HA or a combination injection of BTA and non‐crossed link HA. The type of treatment was randomly selected for each patient from a box of 16 sealed envelopes that contained codes A and B.

To ensure unbiased results, the study was conducted as a double‐blind trial. This means that neither the patient nor the physician who evaluated the clinical images and the statistical expert analyzing the data did not know which treatment method each patient had used. The injections were performed with similar syringes to avoid any potential bias.

## 3 INTERVENTIONS

### 3.1 BTA and crossed link HA combination

Patients in this group received a single injection of a combination of BTA and cross‐linked HA. The injection process involved using Dysport (abobotulinumtoxin A), which was dissolved at 300 units/vial in 2 cc of normal saline. Depending on the extent of the scar and treated area, each volume of Dysport was drawn into a BD luer lock syringe, mixed, and then diluted five times with cross‐linked HA through the interface 30 times. This resulted in each small line of the BD syringe containing 0.6 units of Dysport (microbotax). The cross‐linked HA used had a low G prime of 22 mg NEAUVIA or INTENCE/REOLOGY brand.

Before the injection, local anesthesia was administered using Xyla‐P cream for 45 min. Once the area was numb, it was wiped with an alcohol swab, and a gauge 27 mesotherapy needle was used to inject the solution intradermally under the scars.

### 3.2 BTA and non‐crossed link HA combination

Patients in this group received two injections of a combination of BTA and non‐cross‐linked HA, administered 1 month apart. To prepare for the injection, Dysport (abobotulinumtoxin A) was dissolved at 300 units/vial in 2 cc of normal saline. Depending on the extent of the scar and treated area, each volume of Dysport was drawn into a BD luer lock syringe, mixed, and then diluted five times with non‐cross‐linked HA through the interface 30 times. This resulted in each small line of the BD syringe containing 0.6 units of Dysport (microbotax). The non‐cross‐linked HA used was 532 vials of REVITACARE brand CYTOCARE.

The article "Evaluation and comparison of the efficacy and safety of cross‐linked and non‐cross‐linked hyaluronic acid in combination with botulinum toxin type A in the treatment of atrophic acne scars: A double‐blind randomized clinical trial" was published in 2024. Journal: Skin Res Technol.

Before the injection, local anesthesia was administered using Xyla‐P cream for 45 mins. Once the area was numb, it was wiped with an alcohol swab, and a gauge 30 mesotherapy needle was used to inject the solution intradermally under the scars.

### 3.3 Assessment methods

Follow‐up of patients in each group was performed 3 and 6 months after baseline based on the following description:

1. Evaluation of fine and large pores and spots in terms of number and area,
2. Determination of Goodman and Baron qualitative scar grading system,
3. Determination of patient satisfaction (no response, little, somewhat, good, and excellent), and
4. Recording probable complications.

### 3.4 Statistical analysis

Descriptive statistics including mean [standard deviation (and frequency) (percentage)] was used to analyze continuous and categorical data respectively. To compare continuous and categorical data, an independent‐sample *t*‐test and Chi‐square, or Fisher exact test was used. The one‐way repeated measures ANOVA and Friedman's tests were used to compare continuous and ordinal variables in more than two‐time points. Also, the Marginal Homogeneity or Stuart‐Maxwell test was used to assess changes in paired ordinal data. Statistical significance level was considered at α: 0.05. All data were analyzed using SPSS, version 22.0, Armonk, New York, USA: IBM Corp. Released 2015.

### 3.5 Ethical principles

All information collected was kept confidential and evaluated without a specific name. Participants in this project adhered to all Helsinki ethical principles (IRCT20210718051930N1). This research was approved by the Research Council under the ethics code number IR.IUMS.FMD.REC. 1400.255.

## 4 RESULTS

### 4.1 Basic characteristics

The mean age of patients in the cross‐linked HA and non‐cross‐linked HA groups was 32.75 ± 4.26 and 31.50 ± 8.48 years, respectively, and the difference between the two groups was not statistically significant (*p* = 0.71). Regarding gender, three (37.5%) and seven (87.5%) of the cases in the cross‐linked HA and non‐cross‐linked HA groups, respectively, were female (*p* = 0.11). Further details are shown in Table 1.

**TABLE 1:** Baseline characteristics of included cases (*n* = 16).

		Group		
Variables		Cross‐linked HA *n* (%)	Non‐cross‐linked HA *n* (%)	*p*
Gender	Female	3 (37.5)	7 (87.5)	0.11
Age		32.75 ± 4.26	31.50 ± 8.48	0.71

### 4.2 Comparison of severity outcomes and safety in two groups

#### 4.2.1 Baseline

In the first session, the number of fine pores in the cross‐linked HA and non‐cross‐linked HA groups were 1323.00 ± 485.44 and 923.75 ± 265.05, respectively, and the difference between the two groups was not statistically significant (*p* = 0.05). Also, the area of fine pores in the cross‐linked HA and non‐cross‐linked HA groups was 38 943.38 ± 15 393.03 and 26 205.75 ± 7580.43, respectively (*p* = 0.05). There was also no statistical difference between the two groups in terms of number of large pores, area of large pores, number of spots, and area of spots (Table 2). The acne severity was severe in five (62.5%) and one (12.5%) of the cases in the cross‐linked HA and non‐cross‐linked HA groups, respectively, and this difference was not statistically significant (*p* = 0.08) (Table 2).

The article "Evaluation and comparison of the efficacy and safety of cross‐linked and non‐cross‐linked hyaluronic acid in combination with botulinum toxin type A in the treatment of atrophic acne scars: A double‐blind randomized clinical trial" was published in 2024. Journal: Skin Res Technol.

**TABLE 2:** Comparison of the average of severity score between the understudied groups.

Session	Cross‐linked HA (Mean ± SD)	Non‐cross‐linked HA (Mean ± SD)	*p*
Baseline			
Fine pore count	1323.00 ± 485.44	923.75 ± 265.05	0.05
Fine pore area	38943.38 ± 15393.03	26205.75 ± 7580.43	0.05
Large pore count	532.25 ± 271.85	310.75 ± 114.02	0.06
Large pore area	40148.88 ± 21759.65	23267.13 ± 8760.96	0.05
Spot count	22.25 ± 17.81	15.00 ± 5.45	0.28
Spot area	12528.00 ± 7586.47	14149.63 ± 4543.90	0.61
First follow up			
Fine pore count	1083.88 ± 388.60	808.88 ± 193.55	0.09
Fine pore area	31699.00 ± 11934.72	23109.50 ± 5805.47	0.08
Large pore count	424.38 ± 259.53	264.88 ± 81.55	0.13
Large pore area	32182.25 ± 20304.35	19797.63 ± 5979.81	0.12
Spot count	21.13 ± 15.08	13.75 ± 5.06	0.21
Spot area	14514.25 ± 9954.05	12975.38 ± 5206.88	0.70
Second follow up			
Fine pore count	1009.63 ± 377.71	699.13 ± 217.65	0.06
Fine pore area	29969.50 ± 11550.66	20103.50 ± 6460.78	0.05
Large pore count	521.13 ± 293.29	235.38 ± 73.84	**0.01**
Large pore area	40374.25 ± 23347.76	17723.50 ± 5542.15	**0.01**
Spot count	20.50 ± 11.17	13.63 ± 4.87	0.13
Spot area	13150.25 ± 5561.84	11417.88 ± 5741.58	0.55

### 4.3 First follow‐up session

At the first follow‐up, the number of fine pores in the cross‐linked HA and non‐cross‐linked HA groups was 1083.88 ± 388.60 and 808.88 ± 193.55, respectively, and the difference between the two groups was not statistically significant (*p* = 0.9). Also, the area of fine pores in the cross‐linked HA and non‐cross‐linked HA groups was 31 699.00 ± 11 934.72 and 23 109.50 ± 5805.47, respectively (*p* = 0.08). There was no statistical difference between the two groups in the other indices such as number of large pores (424.38 ± 259.53 vs. 264.88 ± 81.55), area of large pores (32 182.25 ± 20 304.35 vs. 19 797.63 ± 5979.81), number of spots (21.13 ± 15.08 vs. 13.75 ± 5.06), and area of spots (14 514.25 ± 9954.05 vs. 12 975.38 ± 5206.88) (Table 2). The acne severity was moderate in five (62.5%) and three (37.5%) of the cases in the cross‐linked HA and non‐cross‐linked HA groups, respectively, and this difference was not statistically significant (*p* = 0.28). Moreover, none of the patients experienced any adverse effects.

The article "Evaluation and comparison of the efficacy and safety of cross‐linked and non‐cross‐linked hyaluronic acid in combination with botulinum toxin type A in the treatment of atrophic acne scars: A double‐blind randomized clinical trial" was published in 2024. Journal: Skin Res Technol.

### 4.4 Second follow‐up session

After the second follow‐up session, there was a statistically significant difference between the two groups in the number of large pores (521.13 ± 293.29 vs. 235.38 ± 73.84, *p* = 0.01) and the area of large pore (40 374.25 ± 23 347.76 vs. 17 723.50 ± 5542.15, *p* = 0.01). However, there was no statistically significant difference between the two groups in the number of fine pores, area of fine pores, number of spots, and area of spots (Table 2). In the cross‐linked HA group, the acne severity was moderate in two cases (25.0%), while in the non‐cross‐linked HA group, it was moderate in one case (12.5%). However, this difference was not found to be statistically significant (*p* = 0.09). Furthermore, no side effects were observed during this session (Table 3).

**TABLE 3:** Comparison of the acne grade, patients' satisfaction, and side effects between the understudied groups over the time.

Variables	Subgroups	Cross‐linked HA n (%)	non‐cross‐linked HA n (%)	*p*	*p* changes in cross‐linked HA group	*p* changes in non‐cross‐linked HA group
**Acne grade**						
Baseline						
	Macular	0 (0)	0 (0)			
	Mild	1 (12.5)	5 (62.5)			
	Moderate	2 (25.0)	2 (25.0)	0.08		
	Severe	5 (62.5)	1 (12.5)			
First follow up					**0.002**	**0.005**
	Macular	0 (0)	3 (37.5)			
	Mild	3 (37.5)	2 (25.0)			
	Moderate	5 (62.5)	3 (37.5)	0.28		
	Severe	0 (0)	0 (0)			
Second follow up						
	Macular	0 (0)	4 (50.0)			
	Mild	6 (75.0)	3 (37.5)	0.09		
	Moderate	2 (25.0)	1 (12.5)			
	Severe	0 (0)	0 (0)			
**Patients’ satisfaction**						
First follow up						
	No response	0 (0)	1 (12.5)			
	Little	2 (25.0)	3 (37.5)			
	Somewhat	2 (25.0)	3 (37.5)	0.44		
	Good	3 (37.5)	0 (0)			
	Excellent	1 (12.5)	1 (12.5)			
Second follow up					0.31	0.10
	No response	1 (12.5)	0 (0)			
	Little	1 (12.5)	2 (25.0)			
	Somewhat	0 (0)	3 (37.5)	0.22		
	Good	4 (50.0)	3 (37.5)			
	Excellent	2 (25.0)	0 (0)			
Side effects						
First follow up	Yes	0 (0.00)	0 (0.00)			
Second follow up	Yes	0 (0.00)	0 (0.00)	–		

The bold values are statistically significant.

### 4.5 Patient satisfaction

In the comparison of patient satisfaction, the patient's satisfaction level in one (12.5%) of cross‐linked HA and non‐cross‐linked HA groups after the first follow‐up session was excellent (*p* = 0.44). This amount after the second follow‐up session was 2% (25.0%) and 0% in cross‐linked HA and non‐cross‐linked HA groups, respectively (*p* = 0.22). In other words, the level of patient satisfaction among the two studied groups at these times was not statistically significant. Also, the satisfaction level was not significantly changed in both groups over the time (Table 3).

The article "Evaluation and comparison of the efficacy and safety of cross‐linked and non‐cross‐linked hyaluronic acid in combination with botulinum toxin type A in the treatment of atrophic acne scars: A double‐blind randomized clinical trial" was published in 2024. Journal: Skin Res Technol.

### 4.6 Comparison of severity outcomes in two groups over the time

The large pore count decreased from the first session to the last session in cross‐linked HA (from 532.25 ± 271.85 to 521.13 ± 293.29) and non‐cross‐linked HA groups (from 310.75 ± 114.02 to 235.38 ± 73.84). These changes were not statistically significant (*p* = 0.07), but the number of changes in the non‐cross‐linked HA group was significantly higher than in the cross‐linked HA group (*p* = 0.03). Also, the area of large pores increased from the first session to the last session in cross‐linked HA (from 40 148.88 ± 21 759.65 to 40 374.25 ± 23 347.76) and decreased from the first session to the last session in non‐cross‐linked HA groups (from 23 267.13 ± 8760.96 to 17 723.50 ± 5542.15). These changes were not statistically significant (*p* = 0.13), but the number of changes in the non‐cross‐linked HA group was significantly higher than in the cross‐linked HA group (*p* = 0.03), Figure 1.

**FIGURE 1:** Comparison of severity indices in two groups over the time.

The fine pore count decreased significantly from the first session to the last session in cross‐linked HA (from 1323.00 ± 485.44 to 1009.63 ± 377.71) and non‐cross‐linked HA groups (from 923.75 ± 265.05 to 699.13 ± 217.65) (*p* = 0.001), and the number of changes was not statistically significant between the two groups (*p* = 0.06). The area of fine pores decreased significantly from the first session to the last session in cross‐linked HA (from 38 943.38 ± 15 393.03 to 29 969.50 ± 11 550.66) and non‐cross‐linked HA groups (from 26 205.75 ± 7580.43 to 20 103.50 ± 6460.78) (*p* = 0.001), but the number of changes was not statistically significant between the two groups (*p* = 0.06), (Figures 2 and 3).

**FIGURE 2:** The count and area of fine and large pores over the time in the cross‐linked hyaluronic acid group.

**FIGURE 3:** The count and area of fine and large pores over the time in the non‐cross‐linked hyaluronic acid group.

Regarding the acne grade, five (62.5%) and one (12.5%) case had severe grades in the first session in cross‐linked HA and non‐cross‐linked HA groups, respectively. These amounts changed significantly to 0(0%) in the last session for both groups (Table 3). More details are shown in Table 4.

**TABLE 4:** Comparison of the average of severity score between the understudied groups over the time.

Variable	Session	Cross‐linked HA (Mean ± SD)	Non‐cross‐linked HA (Mean ± SD)	*p*	Between‐groups	Time × group	Time
Fine pore count	Baseline	1323.00 ± 485.44	923.75 ± 265.05	0.05	0.06	0.15	**0.001**
	First follow up	1083.88 ± 388.60	808.88 ± 193.55	0.09			
	Second follow up	1009.63 ± 377.71	699.13 ± 217.65	0.06			
Fine pore area	Baseline	38 943.38 ± 15 393.03	26 205.75 ± 7580.43	0.05	0.06	0.12	**0.001**
	First follow up	31 699.00 ± 11 934.72	23 109.50 ± 5805.47	0.08			
	Second follow up	29 969.50 ± 11 550.66	20 103.50 ± 6460.78	0.05			
Large pore count	Baseline	532.25 ± 271.85	310.75 ± 114.02	0.06	**0.03**	0.17	0.07
	First follow up	424.38 ± 259.53	264.88 ± 81.55	**0.011**			
	Second follow up	521.13 ± 293.29	235.38 ± 73.84	**0.01**			
Large pore area	Baseline	40 148.88 ± 21 759.65	23 267.13 ± 8760.96	0.05	**0.03**	0.21	0.13
	First follow up	32 182.25 ± 20 304.35	19 797.63 ± 5979.81	0.12			
	Second follow up	40 374.25 ± 23 347.76	17 723.50 ± 5542.15	**0.01**			
Spot count	Baseline	22.25 ± 17.81	15.00 ± 5.45	0.28	0.19	0.98	0.57
	First follow up	21.13 ± 15.08	13.75 ± 5.06	0.21			
	Second follow up	20.50 ± 11.17	13.63 ± 4.87	0.13			
Spot area	Baseline	12 528.00 ± 7586.47	14 149.63 ± 4543.90	0.61	0.85	0.38	0.54
	First follow up	14 514.25 ± 9954.05	12 975.38 ± 5206.88	0.70			
	Second follow up	13 150.25 ± 5561.84	11 417.88 ± 5741.58	0.55			

The article "Evaluation and comparison of the efficacy and safety of cross‐linked and non‐cross‐linked hyaluronic acid in combination with botulinum toxin type A in the treatment of atrophic acne scars: A double‐blind randomized clinical trial" was published in 2024. Journal: Skin Res Technol.

## 5 DISCUSSION

Acne, characterized as an inflammatory disorder of pilosebaceous units, predominantly affects the younger population, with a higher prevalence among this demographic.^14^ Atrophic facial scarring, a common consequence of acne, poses a significant therapeutic challenge due to its persistent nature and the resulting psychological distress experienced by those affected. Despite the availability of numerous treatments, achieving optimal outcomes often requires multiple interventions for modest improvements. This challenge is compounded by the limited number of prospective clinical trials and comparative studies in this field.^15^

Our investigation explored a novel approach to treating atrophic acne scars using HA gel, specifically in its cross‐linked and non‐cross‐linked forms, combined with botulinum toxin type A. Notably, the application of HA gel, as observed in the study by Hayashi et al.,^16^ proved noteworthy. It demonstrated effectiveness in improving scar appearance and significantly boosted the self‐esteem and self‐confidence of over 80% of the study participants. These findings, corroborated by Reinholz et al.’s research,^17^ underscore the substantial clinical implications of addressing the adverse impact of acne and its associated scars on individuals' quality of life. Given the detrimental impact of acne and its resultant scars on individuals' quality of life, these findings hold significant clinical relevance.

The article "Evaluation and comparison of the efficacy and safety of cross‐linked and non‐cross‐linked hyaluronic acid in combination with botulinum toxin type A in the treatment of atrophic acne scars: A double‐blind randomized clinical trial" was published in 2024. Journal: Skin Res Technol.

Our present study found no significant differences in the count and area of delicate and large pores and spots between the two treatment groups at baseline and in the first follow‐up session. Both methods proved effective for treating acne and related skin conditions (*p* = 0.001). However, during longer‐term follow‐ups, such as at 6 months, combining botulinum toxin and non‐cross‐linked HA emerged as a more practical approach for treating more significant scars.

These observations align with studies by Goodman et al.^18^ and Sherris et al.,^19^ highlighting the multifaceted effects of botulinum toxin in scar management. It is believed to inhibit scar formation, offering a prophylactic advantage in cases involving excisions that may result in scarring that contrasts with relaxed skin tension lines or when revising hypertrophic scars. Furthermore, in the context of existing traumatic or post‐acne scarring, botulinum toxin offers a promising solution for scars in areas prone to exaggeration through movement without inducing untoward cosmetic effects. Importantly, botulinum toxin applications in the upper face regions (forehead, periorbital, glabella) and the lower face areas (chin and its vicinity) have demonstrated efficacy, whether used independently or, more commonly, in conjunction with complementary techniques such as dermal fillers, resurfacing procedures, or surgical interventions,^20^ as demonstrated by studies by Rullan et al.^21^ and Aalami Harandi et al.^22^ The synergistic combination of botulinum toxin with other therapeutic modalities has consistently shown enhanced effectiveness in scar management.

In the research conducted by Joon Seok et al.,^23^ HA filler injections were primarily employed for facial, hand, and neck corrections and enhancements. Due to their established efficacy and painless application, these injections are typically administered using an auto‐seal microneedle intradermal injector. Furthermore, findings from Hai‐yan Cheng's study^24^ revealed that pneumatic injections of non‐cross‐linked HA resulted in significant improvements in skin texture, reduced pore size, and amelioration of fine wrinkles, along with reduced transepidermal water loss (TEWL). Importantly, this treatment approach demonstrated a favorable safety profile, characterized by no complications and downtime, and yielded highly satisfactory results.

In our present study, regarding acne grade, initially, 62.5% of cases in the cross‐linked HA group and 12.5% in the non‐cross‐linked HA group were classified as severe grade. However, in the final session, these percentages markedly decreased to 0% for both groups (*p* = 0.002 and 0.005, respectively).

The article "Evaluation and comparison of the efficacy and safety of cross‐linked and non‐cross‐linked hyaluronic acid in combination with botulinum toxin type A in the treatment of atrophic acne scars: A double‐blind randomized clinical trial" was published in 2024. Journal: Skin Res Technol.

We must acknowledge several limitations of our research, including the relatively small sample size, occasional non‐compliance of some patients with the recommended follow‐up schedule, and the occurrence of treatment complications in the cross‐linked HA group. Notably, two patients in this group experienced the development of multiple subcutaneous nodules during the initial follow‐up session; however, these issues were successfully resolved by the second follow‐up session.

Our study stands out by delving into the uncharted territory of comparing the efficacy of cross‐linked and non‐cross‐linked HA in combination with botulinum toxin type A for treating atrophic acne scars. While botulinum toxin has been approved for atrophic acne scar treatment, our research provides valuable insights into the varying outcomes achievable when used with distinct forms of HA. These findings pave the way for personalized scar management strategies and offer new avenues for advancing the field.

## 6 CONCLUSION

The study conclusively showed that both cross‐linked HA and non‐cross‐linked HA effectively reduced acne severity and enhanced the appearance of pores and spots. Both treatments exhibited comparable effects on fine pores, spots, and overall acne severity. Nevertheless, non‐cross‐linked HA yielded superior results in addressing larger pores than cross‐linked HA.

## CONFLICT OF INTEREST STATEMENT

All authors declare no conflict of interest for this project.

## Data Availability

The data supporting the results of this study are available from the corresponding author.
